This article has been retracted.

# Studying the Role and Molecular Mechanisms of *MAP4K3* in Sorafenib Resistance of Hepatocellular Carcinoma

**DOI:** 10.1155/2020/4965670

**Published:** 2020-11-05

**Authors:** Yi Shi, Xiaofei Mo, Simei Hong, Tianbao Li, Baozhen Chen, Gang Chen

**Affiliations:** ^1^Departments of Molecular Pathology, Fujian Cancer Hospital and Fujian Medical University Cancer Hospital, Fuzhou, Fujian 350014, China; ^2^The School of Basic Medical Sciences, Fujian Medical University, Fuzhou, Fujian 350014, China; ^3^Geneis Beijing Co., Ltd., Beijing 100102, China; ^4^Departments of Pathology, Fujian Cancer Hospital and Fujian Medical University Cancer Hospital, Fuzhou, Fujian 350014, China

## Abstract

Sorafenib is the first FDA-approved therapeutic drug for molecular target medication on advanced-stage hepatocellular carcinoma. It is reported that sorafenib could improve the survival of progression-free patients for 4 to 6 months; however, most of the patients developed drug resistance. Thus, it is critical to reveal the biological mechanisms behind sorafenib resistance. In this study, a sorafenib-resistant model was developed by exposing HepG2 cells to sorafenib with gradient increasing concentration, and the resistance-related genes were screened by microarray. Real-time qPCR was used to validate selected gene expression of the resistance model, and lentivirus vector-mediated RNA interference was applied for specific gene knockdown. In addition, high-throughput High Celigo Select (HCS) and flow cytometry were used to measure the effect on cellular proliferation and apoptosis. As a result, our study established a sorafenib-resistant model with IC_50_ of 9.988 *μ*M. The Affymetrix expression profile of the sorafenib-resistant model showed 35 resistant-related genes, and 91.4% of the resistant genes showed upregulation in HepG2 resistance cells. In addition, 20 genes were knocked down to measure cell proliferation, and *MAP4K3* with high proliferation inhibiting phenotype was chosen for further study. Meanwhile, the HCS results revealed that shMAP4K3 transfection could downregulate resistant cell proliferation, and the flow cytometry results showed that cell apoptosis was significantly increased in the *MAP4K3* knockdown group. In summary, *MAP4K3* is a novel molecular marker for improving the drug sensitivity of sorafenib treatment in hepatocellular carcinoma.

## 1. Introduction

Liver cancer (LC) ranks fifth in frequency in the world. The numbers of annual cases and deaths of LC are 460,000 and 420,000, respectively, accounting for 10.9% cancer incidence and 15.0% cancer mortality in China [1]. Hepatocellular carcinoma is the most common pathological type of liver cancers with approximately 70% to 90% incidence of the primary liver cancer being hepatocellular carcinoma. Sorafenib was first approved as a small molecular target medication targeting serine/threonine and tyrosine kinase receptor and marketed as Nexavar for treatment of advanced-stage hepatocellular carcinoma (HCC). Previous molecular studies revealed that sorafenib showed antitumor effects by blocking cell proliferation through inhibiting Raf kinase, VEGF1-3, and PDF receptor, and sorafenib has been approved as the first-line drug of systematic treatment for advanced hepatocellular carcinoma [2, 3]. Two important phase III clinical trials conducted by Tremosini et al. and Rosell et al. showed that sorafenib significantly improved the overall survival (OS) in advanced hepatocellular carcinoma patients by 44% and 47%, while time to progression (TTP) was improved by about 73% and approximately onefold, respectively [4, 5]. Besides the improvement of OS and TTP, sorafenib could decrease the risk of macrovascular infiltration and extrahepatic metastasis, regardless of patients with advanced HCC having macrovascular infiltration and extrahepatic metastasis or not. Recent studies suggested that sorafenib significantly improved OS and TTP in patients with hepatocellular carcinoma resulting from alcoholic liver disease [6]. In another subtype study, sorafenib combined with TACE also achieved promising results; TTP was improved by 10.6 months, along with the improvement of median progression-free survival and median survival time. The combination of sorafenib and other chemotherapy drugs, including gemcitabine, doxorubicin, fluorouracil, and oxaliplatin, also achieved well treatment efficacy in clinical practice [7, 8]. Moreover, sorafenib could be applied for preventing recurrence of patients after liver transplantation as well [9].

Although sorafenib has good treatment efficacy, resistance during treatment limits the usage in clinical application. Patients initially respond to sorafenib well and have an improved clinical outcome for about 4 to 6 months; however, all of them developed progression after that [10]. No specific molecular markers were found to predict the sensitivity of clinical treatment, and the resistant mechanism of sorafenib is still uncertain. Moreover, the underlying molecular mechanism of development and progression of hepatocellular carcinoma is complicated and could not explain the mechanism of sorafenib resistance in clinical practice.

In summary, our study is aimed at investigating the molecular mechanism of sorafenib resistance in hepatocellular carcinoma by constructing a sorafenib-resistant model of the HepG2 cell. Moreover, we found novel molecular markers to predict efficacy and sensitivity of treatment. Our study provided a novel approach for exploring sorafenib sensitivity and to overcome its resistance in clinical practice.

## 2. Materials and Methods

HepG2 resistance cells were constructed by the concentration gradient method. CellTiter-Glo Luminescent Cell Viability (Promega) was used to measure the activity of HepG2 control/HepG2 resistance cells and validate whether the HepG2 resistance cells are resistant to sorafenib by measuring cell activity with a specific concentration of sorafenib. Affymetrix expression profile microarray was performed to screen drug-resistant genes in HepG2 resistance cells. The selection criteria were as follows: the screening standard was considered as log2 fold change over 2 and *P* value less than 0.05 compared with the HepG2 control group. Applying bioinformatics analysis, 35 upregulated resistance-related genes were selected for further experiments. Highly expressed genes in drug-resistant strains were considered primarily malignant, while relatively low expressed genes were suppressed. A real-time qPCR technique was applied to evaluate the endogenous gene expression in HepG2 resistance cells. Among 35 resistant-related genes, there were 32 highly expressed resistance-related genes in HepG2 resistance cells, and 20 of these genes were randomly selected. High-throughput High Celigo Select (HCS) was applied to evaluate the effect on proliferation after gene knockdown.

The shRNA plasmid vector with interference *MAP4K3* gene was constructed for lentivirus infection. The lentivirus with *MAP4K3* shRNA was infected into HepG2 and sorafenib resistance cell lines to generate stable knockdown cell lines. The infection condition included enhanced infection solution (EN.iS) with polybrene, and the fluorescence was observed after 72 hours. Flow cytometry was used to measure the cell apoptosis and cell count at each stage of the cell cycle for primarily investigating the *MAP4K3* gene function and the underlying mechanism of sorafenib resistance in hepatocellular carcinoma.

## 3. Results

The IC_50_ of HepG2 control cell and HepG2 resistance cell were measured with an increasing dose of sorafenib. The proliferation inhibition of HepG2 control cell was significantly increased; however, the proliferation inhibition of HepG2 resistance cells showed no significant difference before 10 *μ*M, which proved that the selected HepG2 resistance strain was indeed resistant to sorafenib (Figure 1).

### 3.1. Affymetrix Expression Profile for Drug-Resistant Gene Screening

The volcano plot showed the distribution and scatter plots. The selection criteria of significant expression were set as follows: fold change more than 2 and *P* value less than 0.05. The results showed that compared with HepG2 cells, 295 upregulated genes and 211 downregulated genes were differently expressed in the HepG2 resistance group (Figure 2(a)). The heat map showed the distribution of the top 35 differential genes between the control group and the sorafenib-resistant group. Each entry in Figure 2(b) denoted the log2 expression of genes in the corresponding sample, with red being positive and blue being negative (Figure 2(b) and Supplementary Figure 1).

### 3.2. Real-Time qPCR Validation

Real-time qPCR technique was used to study 35 drug-resistant endogenous gene expression in HepG2; therefore, 32 drug-resistant genes were confirmed with high expression in HepG2 resistance cells (Figure 3). Among 32 high-expressed genes, 20 genes were selected by high-throughput High Celigo Select (HCS) through comparison of knockdown efficiency of proliferation (Supplementary Figure 2). *MAP4K3* is one of the critical genes with a high proliferation-inhibiting phenotype and was confirmed by qPCR as differentially expressed genes between drug resistance and normal control cell lines; therefore, *MAP4K3* gene was selected for further study.

### 3.3. *MAP4K3* Inference Sequence Infected Resistance to Sorafenib

We applied a fluorescence scope to check the infection efficiency of *MAP4K3* knockdown, and the results showed that the infection efficiency was reaching 80%, indicating that lentivirus successfully infected HepG2 with RNA interference sequence of the target gene (Figure 4).

### 3.4. *MAP4K3* Affects the Proliferation of HepG2

Within the HCS results, three siRNAs targeting *MAP4K3* were transfected into HepG2 cells together and the cell proliferation was significantly inhibited over 50% after 5 days in *MAP4K3* knockdown cell lines. Meanwhile, compared with the control group, the knockdown efficiency of different siRNAs (*MAP4K3-1*, *MAP4K3-2*, and *MAP4K3-3*) was 68.5%, 57.6%, and 59.4% by qPCR, respectively, and the difference was statistically significant (*P* < 0.05), indicating that *MAP4K3* gene had been successfully knocked down (Figure 5).

### 3.5. Apoptosis and Cell Cycle Analysis

Compared with the control (shCtrl), the sh*MAP4K3* group showed that cell apoptosis is significantly increased in sh*MAP4K3* (*P* < 0.05), and the difference was statistically significant. This result also indicated that *MAP4K3* was significantly associated with cell apoptosis in HepG2 resistant to sorafenib strain (Figure 6(a)). The cell cycle assay showed that cell counts in the HepG2 resistance group with knockdown of *MAP4K3* was decreased in the G2/M stage; however, cell counts increased on the G1 stage (Figure 6(b)). Compared with the control group, apoptosis and cell cycle experiments revealed that cells at G1 and G2/M stages in the KD+sorafenib group showed significantly different by *t*-test analysis (*P* < 0.05). However, there was no significant difference between groups at the S stage by *t*-test analysis (*P* > 0.05) (Figure 6(c)).

## 4. Conclusion

This study for the first time investigated the relationship between *MAP4K3* gene and sorafenib resistance in hepatocellular carcinoma as well as explore potential underlying molecular mechanisms. We identified that *MAP4K3* is the key drug resistance relative gene in hepatocellular carcinoma and provide an experimental basis for seeking biomarkers to develop effective therapy for patients who are not qualified for surgical intervention.

## 5. Discussion

There are two methods which are widely used to conduct the drug resistance models, including the high-dose intermittence method and the concentration gradient method [11]. The advantage of the concentration gradient method is that the drug dose is gradually increased, with extraenvironmental changes of cell culture which are gradually changed, and cells are easy to tolerate and maintain in good status. Sorafenib is an oral multikinase inhibitor which can inhibit cancer cell proliferation and angiogenesis, as well as promote cancer cell apoptosis. And sorafenib requires long-term oral taking to maintain the blood concentration; therefore, the concentration gradient method is relatively suitable to conduct our drug resistance model. In this study, we aimed to explore the underlying mechanism of sorafenib resistance by using the concentration gradient method to conduct the drug resistance model.

There are many methods to evaluate the cell resistance model, including proliferation and apoptosis as well as resistant-relative protein assay such as MDR, Pgp, and GST [12, 13]. In our study, the resistance cell line was evaluated by the cell shape and survival status: firstly, cells could survive in high drug concentrations of drugs and still maintain relatively good status during the process of changing the sorafenib concentration. Secondly, inhibition of half counts (IC_50_) was calculated as tolerance ability, and higher IC_50_ indicated the cells showing higher resistance to sorafenib. Meanwhile, the resistance index (RI) is calculated spontaneously, and RI equals to IC_50_ of resistance cells over parental cells. Our study showed that the IC_50_ of HepG2 cell is 1.672 *μ*M, and with increased sorafenib concentration, the status of HepG2 resistance cells was significantly worsened and the resistant activity of HepG2 cells continued to rise. While HepG2 resistance cells could grow stably in 5 *μ*M of sorafenib culture with good shape and status, the IC_50_ of HepG2 resistant to sorafenib was 9.988 *μ*M, which was consistent with previous literature reported [14–16]. The resistance index (RI) was 5.97, which is relatively higher. Therefore, we have evidences to believe that the screened out HepG2 cells were resistant to sorafenib.

Sorafenib has well-known pharmacological function, and the drug resistance studies have been focusing on its pharmacological-related signal pathways. Sorafenib works primarily on two resistance pathways: it can directly inhibit tumor cell proliferation through *Ras/Raf/MEK/ERK*, *PI3K/Akt*, and *JAK/STAT* signaling pathways; on the other hand, it suppresses angiogenesis through vascular endothelial growth factor receptor (*VEGFR*) and platelet-derived growth factor receptor (*PDGFR*) as well. The *MAPK* signaling pathway has been widely reported in the initiation and development of hepatocellular carcinoma as well as its application in the clinical practice. *MAP4K3* can be activated by extracellular stimuli, mediating signaling from the cellular membrane to nuclei transduction through *MAP4K3* cascade pathways of multiple protein kinases. *MAP4K3* participates and regulates the biological process of cell survival, growth, development, proliferation, differentiation, autophagy, and apoptosis [17]. Numerous studies have reported that *MAP4K3* overexpression occurs in cancer tissues of hepatocellular carcinoma as well as in other cancers [18, 19]. The upregulation of *MAP4K3* is correlated with cancer recurrence and induces cell migration and promotes cancer metastasis and invasion. Recent studies revealed the potential mechanisms of *MAP4K3* with cancer metastasis and recurrence; *MAP4K3* could promote distant metastasis instead of initiating tumorigenesis in the animal study. There are also studies reporting that *MAP4K3* overexpression may contribute to metastasis through proinflammatory pathways or environmental changes.

Studies reported that c-Jun N-terminal kinase (*JNK*), another *MAPK* family member, could serve as a biomarker to predict the cell sensitivity to sorafenib. The effect of *JNK* on the initiation and development has also been reported in hepatocellular carcinoma. Sun et al. reported that melatonin combined with sorafenib could inhibit hepatocellular carcinoma cell growth and promote apoptosis through the *JNK* signaling pathway [20, 21]. The *JAK/STAT3* signaling pathway promotes antiapoptosis protein such as *Mcl-I* and *cyclin D1* transduction. The upregulated *JNK* pathway played a critical role in the initiation and development of hepatocellular carcinoma. Overall, the *JNK* signaling pathway is highly associated with the sensitivity of sorafenib in hepatocellular carcinoma cells [22].

The hepatocellular carcinoma is a solid tumor; therefore, the tissue angiogenesis plays a critical role in hepatocellular carcinoma growth and invasion. Studies have shown that the proliferation, migration, and adhesion of endothelial cells in hepatocellular carcinoma were different in terms of gene expression and pathological process from normal tissue. Although sorafenib plays an important role in improving patient survival time in patients with hepatocellular carcinoma, its efficacy has been questioned due to developing resistance in a short time. The mechanism of resistance is also implicated in the reduction of tumor cell sensitivity to sorafenib epithelial-mesenchymal transduction (EMT) or sensitivity to hypoxia-induced response [23, 24].

This study has successfully constructed a HepG2 resistant to sorafenib model, used Affymetrix expression profile microarray analysis, and applied HCS to select highly expressed gene—*MAP4K3*. We did find out that *MAP4K3* has effects on cellular proliferation, apoptosis, and cell cycle, which can potentially explain the *MAP4K3* roles in resistance. Further studies are needed to investigate the roles of the *MAP4K3* gene in multiple pathways by the HepG2 resistance model.

## Figures and Tables

**Figure 1:** HepG2 resistant to sorafenib model.

**Figure 2:** Affymetrix expression profile microarray analysis. (a) The *x*-axis indicated the sorafenib-resistant group, and the *y*-axis indicated the control group. (b) The heat map showed the significant differentially expressed genes between the drug-resistant (DR) group and the normal control (NC) group.

**Figure 3:** Amplification curve of endogenous drug-resistant gene expression which was measured by real-time qPCR technique. Among 35 drug-resistant genes which were selected by Affymetrix expression profile, real-time PCR was not performed on number 13 *SEMA3G* gene and number 19 *HIST1H2BC* gene due to difficulty of primer design. Except for number 23 *PTPTN2* gene with low abundance, the remaining 32 drug-resistant genes have high abundance.

**Figure 4:** HepG2 of lentivirus with *MAP4K3* inference sequence infected resistance to sorafenib: (a) the clear field view of shCtrl cells; (b) fluorescence field view of shCtrl cells; (c) the clear view of sh*MAP4K3* cells; (d) the fluorescence field view of sh*MAP4K3* cells, indicating lentivirus successfully infected HepG2 containing *MAP4K3* RNA interference sequence.

**Figure 5:** The process of drug-resistant gene. (a) The fold of cell proliferation of sh*MAP4K3* knockdown compared with the shCtrl group at different time points. (b) The knockdown efficiency of shRNA of *MAP4K3-1*, *MAP4K3-2*, and *MAP4K3-3*, respectively.

**Figure 6:** (a) Apoptosis analysis of RNA lentivirus infected HepG2 with sorafenib treatment. (b) Cell cycle analysis of *MAP3K4* knockdown cell lines with sorafenib. (c) Histogram results of the flow cytometer for cell cycle counts.

## Data Availability

The data of this study are available from the corresponding author upon request.

## Supplementary Materials

Supplementary Materials Supplementary Figure 1: gene enrichment in empiric signaling pathway. Supplementary Figure 2: the proliferation efficacy of 20 selected genes knocked down.
